# Exosome-delivered BMP-2 and polyaspartic acid promotes tendon bone healing in rotator cuff tear via Smad/RUNX2 signaling pathway

This article has been retracted.

**DOI:** 10.1080/21655979.2021.2019871

**Published:** 2022-01-04

**Authors:** Lei Han, Hong Liu, Huajun Fu, Yugen Hu, Weili Fang, Junsheng Liu

**Affiliations:** Department of Orthopaedics Institute, Xiaoshan Traditional Chinese Medical Hospital, Hangzhou, Zhejiang, China

**Keywords:** Rotator cuff injury, tendon bone healing, BMP-2, Smad/RUNX2, signaling pathway

## Abstract

Rotator cuff tear is the main form of shoulder joint injury, which seriously affects shoulder joint function. This study aimed to clarify the function and mechanism of exosomes containing polylactic acid (PLA), polylactic acid copolymer and BMP-2 in tendon bone healing of rotator cuff tear. First, CD44 expression in bone marrow mesenchymal stem cells (BMSCs) and CD90 and CD44 in exosomes were analyzed by flow cytometry. Then, stability and targeting identification of exosome-delivered bone morphogenetic protein (BMP)-2 and PLA microcapsules were measured by transmission electron microscopy (TEM), DiO/DiI staining. Finally, tendon-bone repair after acute rotator cuff rupture in rabbits was established, and the function of BMP-2 exosomes for tendon bone healing in rotator cuff tear was evaluated by micro-CT, biomechanical determination and histochemical staining methods. The results showed that the exosomes of polyaspartic acid-polylactic acid-glycolic acid copolymer (PASP-PLGA) microcapsules were successfully established which showed good stability and targeting. The bone mineral density (BMD), tissue mineral density (TMD) and bone volume fraction (BV/TV) were higher, while the stiffness and the ultimate load strength of the tendon interface were enhanced under treatment with exosomes of PASP-PLGA microcapsules. Histochemical staining showed that exosomes of PASP-PLGA microcapsules promoted tendon and bone interface healing after rotator cuff injury. The tendon regeneration- and cartilage differentiation-related protein expressions were significantly upregulated under treatment with exosomes of PASP-PLGA microcapsules. In conclusion, exosome-delivered BMP-2 and PLA promoted tendon bone healing in rotator cuff tear via Smad/RUNX2 pathway. Our findings may provide a new insight for promoting tendon healing.

## Introduction

Rotator cuff injury is a common disease in sports medicine, which leads to shoulder joint pain and dysfunction [1]. So far, the clinical measures used for the treatment include physical therapy, such as light, electricity, and heat [2,3]. Recently, great improvements have been made in the treatment of rotator cuff repair, including manual rehabilitation, intra-articular injection of drugs, surgical treatment, etc., as well as some emerging technologies. However, repair failures remain frequently obscure owing to the size of the tear, the difference in repair technology, and the postoperative rehabilitation [4]. Therefore, the treatment of rotator cuff injury is still a clinical problem. Firm tendon–bone interface healing can buffer the induction force and reduce the occurrence of tearing [5]. It has become a prerequisite for ligament reconstruction and rotator cuff repair to exert its physiological. However, the tendon–bone interface is difficult to heal.

Mesenchymal stem cells differentiating into cartilage can promote the regeneration of cartilage at the tendon–bone interface during the healing process of the rotator cuff, making it possible to restore the tissue performance at the tendon-bone junction by synthesizing the cartilage matrix [6]. Transforming growth factor is a kind of endogenous biological polypeptide, which can stimulate cell growth and differentiation, cartilage synthesis, and regeneration of damaged cartilage tissue [7,8]. Bone morphogenetic protein (BMP), which belongs to the family of transforming growth factors, is the only growth factor that can induce bone tissue formation alone. Of them, BMP-2 is an effective inducing factor for the growth and differentiation of osteogenic and chondrogenic cells [9]. However, it seriously limits the application of BMP-2 in the treatment of rotator cuff injury tendon–bone interface healing because of low content, high acquisition cost and insufficient sustainability in natural bone tissue. It has been demonstrated that it can increase the amount of new bone formation and improve the biomechanical strength by using injectable calcium phosphate cement (CPC) as a carrier to inject recombinant human BMP-2 into the tendon–bone interface of the rabbit anterior cruciate ligament reconstruction model [10]. However, it will cause a series of complications owing to much higher physiological level and the unreasonable release kinetics, such as local soft tissue edema, heterotopic ossification, bone resorption around the implant [11,12]. Therefore, it is necessary to solve the problems of carrier, optimal dose, and effective time of growth factor release in the human body if BMP-2 is widely used in the treatment of clinical rotator cuff injuries.

Exosomes can be secreted by various kinds of cells that can deliver mRNA, miRNA, proteins and other substances secreted by donor cells to recipient cells, thereby realizing information transmission and material exchange between cells [13]. At present, exosomes that have the advantages of low adverse immune response, good blood stability, and high delivery efficiency in drug delivery have been developed as a variety of drug carriers, such as anti-tumor, anti-inflammation, proteins, and genetic drugs [14]. There are also some studies focusing on the application of exosomes to bone growth and metabolism. For instance, Cui et al. have found that macrophage-derived miRNA-containing exosomes induce peritendinous fibrosis after tendon injury through the miR-21-5p/Smad7 pathway [15]. Wei et al. have used BMP-2 to stimulate mesenchymal stem cells to extract exosomes and integrated the exosomes into titanium oxide nanotube biomaterials for research, and they found that this new compound significantly increases the expression of early osteoblast-related markers, activates cell autophagy and promotes bone formation [16]. In addition, polyaspartic acid (PASP) is a kind of artificial biomimetic synthetic polymer material. It can be combined with the active components of some drugs by carboxyl groups on its surface to obtain a more efficient drug loading system. For instance, Xu et al. have synthesized a new type of polyaspartic acid material, which can form polyaspartamide derivative nanoparticles with tunable surface charge that can achieve highly efficient cellular uptake and low cytotoxicity [17]. Recent studies have found that a three-dimensional hydrogel composed of BMP-2 core sequence oligopeptides, phosphoserine, synthetic cell adhesion peptides and polyaspartic acid has bone targeting properties and can synergistically promote bone regeneration by promoting the adhesion and proliferation of bone marrow mesenchymal stem cells in rats [18].

These reports provided the foundation for treating rotator cuff injury, combining the bone targeting properties of polyaspartic acid with the carrier function of exosomes. BMP-2 participates in tendon-bone healing and its function involves its downstream signal transduction mediators, Smad [19]. We wondered whether this signaling involved in tendon bone healing in this research. Therefore, in the present study, we intended to investigate the function and the mechanism of exosomes with PASP carrying polylactic acid-glycolic acid copolymer (PLGA) microcapsules for sustained release of BMP-2 to tendon bone healing in rotator cuff tear. It will not only provide a new idea for promoting tendon-bone healing but also provide the basis for the clinical application.

## Materials and methods

### Isolation, culture and identification of rabbit bone marrow mesenchymal stem cells (BMSCs)

A 4 mL of bone marrow fluid was drawn from tibial in a 3-month-old big-eared white rabbit by a 10-mL syringe (containing 0.5 mL of 2500 U/mL heparin sodium) connected with a bone marrow puncture needle (NO.16). And then the bone marrow fluid was mixed with 4 mL of Dulbecco’s modified Eagle’s medium (DMEM, 12430054, Gibco, USA) supplemented with 10% fetal bovine serum (FBS, Gibco, USA) and centrifuged at 1000 rpm for 20 min. Cells were resuspended and transferred to another sterile centrifuge tube containing 2 times the volume of the lymphocyte separation solution. Subsequently, the cells were centrifuged at 2000 rpm for 20 min, the milky layer liquid was aspirated, and then diluted again, and centrifuged at 1000 r/min for 5 min. The supernatant was discarded. The cells were resuspended, and 1 × 10^6^ cells/mL were cultured in the 90% DMEM medium supplemented with 10% FBS, 100 μg/mL penicillin and 100 μg/mL streptomycin at 37°C in a 5% CO_2_-contained incubator under 95% saturation humidity. Subculture was performed when the cell confluence reached 80%. Cell purity identification was detected by cell morphology observation under the microscope, and CD44 expression was determined by flow cytometry analysis. All the experiments were approved by the Ethics Committee of Xiaoshan Traditional Chinese Medical Hospital. The contents of this study were under full compliance with government policy and the Declaration of Helsinki.

### Flow cytometry analysis

BMSCs were detached with 0.25% trypsin-EDTA (Gibco) for 20–30 s and centrifuged at 1000 rpm for 5 min. After the supernatant was removed, cells were washed twice by PBS, and then, they were collected and resuspended in PBS. Cell surface markers, CD90-FITC and CD44-FITC, were used to label the cells on ice for 30 min in the dark. Cell suspensions without the antibodies served as controls. Cells were washed twice and resuspended in 200 μL of PBS before analysis. All antibodies were purchased from BD Biosciences. Flow cytometry was performed with a flow cytometer (Beckman Coulter).

### Extraction and identification of exosomes from BMSCs

Exosomes from BMSCs were extracted by Total Exosome Isolation Reagent (from cell culture media) (4478359, Thermo Fisher, USA). Morphology of exosomes was identified by transmission electron microscopy (TEM). Briefly, exosomes were diluted to 500 μg/mL and fixed with 2.5% glutaraldehyde for 2 h. The 20 μL of fixed exosomes were taken to the copper mesh, and it was dried under an infrared lamp for 30 min. Then one drop of 1% phosphotungstic acid solution with pH 6.8 was added and dyed for 5 min. The exosomes morphology was observed and imaged under TEM (HT7700; HITACHI, Tokyo, Japan) at 80 kV. Nanoparticle tracking analysis (NTA) was detected by NanoSight NS300 (Malvern, England). The diameter and concentration were calculated by Stocker-Einstein equation: D*VIS = kT/6*PI*R.

### Preparation of PLGA microcapsules encapsulating BMP-2

BMP-2 was dissolved in 200 μg of distilled water and mixed with dichloromethane dissolved with PLGA and emulsifier uniformly. Subsequently, the mixture was treated ultrasonically for 20 min to form an initial emulsion. The initial emulsion was dropped into 40 mL of different concentrations of polyvinyl alcohol (PVA) solution and ultrasonically emulsified for 10 min to form a double emulsion. The microcapsules were centrifuged repeatedly at 8000 rpm for 10 min, washed three times, collected, and freeze-dried overnight. The microcapsules were sealed, dried, and stored in a refrigerator at −20℃ for further use. A 20 mg of microcapsules was suspended in PBS (pH 7.4), and the sample was placed in a constant temperature shaking box and shaken for 36 h under 37°C at 100 rpm. Then, the sample was centrifuged, and the supernatant was collected. The concentration of BMP-2 in the supernatant was measured by a Human BMP-2 ELISA kit (ab277085, Abcam, UK) to calculate the amount of microencapsulated BMP-2. The microencapsulation rate was calculated by the following formula: EE (%) = encapsulated BMP-2/invested BMP-2×100%.

### Preparation of polyaspartic acid (PASP) short peptide gel and PLGA-PASP microcapsules

A mixture of PASP short peptide KIPKASSVPTELSAIS and phosphoserine was biosynthesized. The 0.5 mg of the mixture was dissolved in 1 mL of deionized water to obtain a nanoparticle solution overnight. The 25 μL of nanoparticle solution (30 mg/mL), 25 μL of sodium alginate (10 mg/mL) and 25 μL of calcium oxide solution (2 mol/L) were mixed in deionized water at room temperature to obtain an active hydrogel. Finally, PLGA-PASP microcapsules were prepared by using the dichloromethane fumigation method. Briefly, the microcapsules were directly fused into a porous scaffold material and mixed with polyaspartic acid peptide under vacuum conditions and the polyaspartic acid peptide gel was absorbed into the pores of the microcapsule support and the combination was completed. All tests were repeated three times in triplicate.

### Stability and targeting identification of exosome-delivered BMP-2 and polyaspartic acid microcapsule

PLGA-PASP microcapsules and exosomes were co-incubated for 2 h at room temperature to form exosome-delivered BMP-2 and polyaspartic acid microcapsule. The morphological changes of exosomes were identified by transmission electron microscopy (TEM). Exosome markers, Alix and Annexin V, a marker for contamination, Calnexin, as well as the loading control, GAPDH, were also detected by Western blot. Targeting analysis was performed using DiO and DiI staining. Control group was untreated cells, Control-Exo goup was exosomes treated with sEVs only, Blank-Exo group was exosomes treated with empty microcapsules, and BMP-2-Exo group was exosomes with BMP-2-loaded microcapsules and sEVs. Lipophilic tracers such as DiO (Invitrogen, Carlsbad, CA, USA; green fluorescence) and DiI (red fluorescence) were prepared in stock solutions in dimethylsulfoxide (DMSO). Briefly, BMSCs (1 × 10^5^ cells/mL) and exosome-delivered BMP-2 and PLA microcapsules (100 μg/mL) were staining by DiO or DiI fluorescent dyes (1 μM) at 37°C for 15 min, respectively. Then, BMSCs and exosomes were co-incubated for 1, 2 and 3 h, respectively. Finally, the BMSCs were detected by fluorescent microscopy at 484 nm and 549 nm, respectively. Fluorescence signals were quantified using the ImageJ software.

### Establishment of rabbit models of tendon-bone repair after acute rotator cuff rupture

A total of 27 big-eared white rabbits were used to establish a model for tendon-bone repair after an acute rotator cuff rupture. In addition, another three big-eared white rabbits were used as control with MRI examinations on bilateral shoulder joints. Briefly, sumianxin II (0.2 mL/kg) was injected intramuscularly into the 27 big-eared white rabbits for general anesthesia. After being successfully anesthetized, they were placed in a prone position. A longitudinal skin incision approximately 2 cm in length was made at the shoulder joint, and the deltoid muscle was separated bluntly. At the stop point of the large nodule, the supraspinatus tendon was sharply cut, and a 0.5 cm × 0.5 cm tendon tissue was removed to create a full-thickness rotator cuff injury model. The tendon-bone suture was performed to reconstruct the supraspinatus tendon attachment point. The joint cavity and subcutaneous were washed with gentamicin saline with no active bleeding, muscle bonds broken and sutured correctly. The animal model was fixed in plaster after the operation, and 200,000 U of penicillin was routinely injected intramuscularly, twice daily, for 3 days. During the plaster fixation period, the diet was assisted artificially, and the plaster was removed after 1 week. After the animal modeling was completed (on the day of the surgery), 27 rabbits were randomly divided into 3 groups (n = 9 each group) by injection with different exosomes into the key bone interface, including Control-Exo, Blank-Exo, and BMP-2-Exo groups. MRI and CT scan were performed to evaluate the tendon-bone complex repair process and the formation of bone structure at the tendon–bone interface at 6, 12, and 18 weeks after the operation before the histological observation. Bone quality at the SSp tendon insertion on the greater tuberosity was assessed with micro-CT (Explore CT-120; GE Healthcare, London, Ontario, Canada) at a resolution of 50 mm, 100 kV, and 50 mA. Acquired images were processed with MicroView2.2 (GE Healthcare). The region of interest (ROI) included the greater tuberosity proximal to the humeral growth plate. Bone mineral density (BMD), tissue mineral density (TMD) and bone volume fraction (BV/TV) were evaluated.

### Biomechanical determination

The shoulder joint specimens from different groups were collected at 12 weeks after the operation to determine the biomechanical properties of the tendon-bone complex after the operation of the animal model. Six samples from each operating group were used for biomechanical analysis. In brief, all soft tissues except for the reconstruction of the supraspinatus tendon stop and the tendon-bone structure were removed and stored at −80°C. The lateral width of the rabbit supraspinatus tendon was measured with a vernier caliper, and then the middle thickness of the tendon was measured with a measuring instrument, and the cross-sectional area of the rabbit supraspinatus tendon was calculated. Stretching test was performed by the MTS858 biomaterial testing machine. The length of the rabbit supraspinatus tendon was measured with an electronic vernier caliper when the tension reached 2.0 N. Pre-treatment was performed with a tensile speed of 0.5 mm/s and an elongation of 0.5 mm for 3 times, and then a tensile breaking test was performed at a tensile speed of 500 mm/min. The testing machine drew a load–displacement curve and carried out the maximum load, and biomechanical indexes of stiffness, and maximum strength were calculated.

### Histochemical staining analysis

Tissue specimens from different groups were obtained and sliced into 4-μm sections followed by embedding in paraffin used for histochemical staining, including hematoxylin–eosin (HE), Alcianblue and Masson staining. For HE staining, deparaffinized sections were stained in a hematoxylin staining solution for 3–5 min and followed by differentiation, returned blue and rinsed with running water. The slices were dehydrated with 85% and 95% gradient alcohol for 5 min, respectively, and stained in an eosin staining solution for 5 min. Dehydrated and sealed, the slides were dehydrated and sealed with neutral gum. For Masson staining, the slices were soaked by Masson A solution overnight, and washed with tap water. And then slides were soaked for 1 min with dye solution of Masson B solution and Masson C solution in equal proportion followed by differentiation with 1% hydrochloric acid alcohol. Masson D solution was used to incubate the slices for 6 min and immersion into the Masson E and Masson F solution for 1 min and 2–30 s, respectively. For Alcianblue staining, the slices were stained with Alcian Blue (PH = 2.5) solution for 30 min at room temperature, and then the slides were washed in running tap water for 5 min and rinsed in DI water. Subsequently, the slides were counterstained in a nuclear fast red for 5 min at room temperature. Finally, the slides were washed three times in DI water. The tissue slices were taken by a microscope (Olympus, Japan).

### Western blotting

Total protein was extracted from tissues and HK-2 cells using RIPA Lysis buffer (P0013, Beyotime, Shanghai, China) with 1 mM of PMSF following the manufacturer’s instructions. Proteins were quantified using the BCA™ Protein Assay Kit (Biosharp, BL521A). The 30 g of proteins were boiled at 100°C for each sample with protein loading buffer for 5 min, followed by separation in 10–12% SDS-PAGE electrophoresis and transferred onto PVDF membranes. Then, 5% lipid-free milk/TBST buffer was used to block the membranes at room temperature overnight, and incubated with primary antibodies of anti-Alix (ab27537, 1:1000, Abcam), anti-Annexin V (ab14196, 1:1000, Abcam), anti-TSG101 (ab125011, 1:1000, Abcam), anti-Calnexin (ab133615, 1:1000, Abcam), anti-CBFβ (ab111577, 1:1000, Abcam), anti-TGFβ (ab215715, 1:1000, Abcam), anti-Smad3 (ab40854, 1:1000, Abcam), anti-Smad4 (ab230815, 1:1000, Abcam), anti-Smad5 (ab40771, 1:2000, Abcam), anti-RUNX1(ab240639, 1:3000, Abcam), anti-RUNX2 (ab192256, 1:2000, Abcam), anti-Notch3 (ab23426, 1:1500, Abcam), anti-Aggrecan (ab3778, 1:1000, Abcam), anti-Collagen II (ab188570, 1:5000, Abcam), anti-SOX-9 (ab185966, 1:5000, Abcam), anti-TIMP-1 (ab211926, 1:5000, Abcam) and anti-GAPDH (ab8245, 1:5000, Abcam) for 2 h at 4°C overnight, respectively. After incubated with secondary antibodies anti-mouse IgG (BA1051, 1:10000, BOSTR) or anti-rabbit IgG (BA1054, 1:15000, BOSTR) for 1–2 h at room temperature, the immuno-complexes were finally detected by ECL after washing by TBST and analyzed using the Image-Pro Plus 6.0 software.

### Statistical analysis

Data were shown as the mean ± standard deviation from at least three independent experiments. Statistical comparisons were performed using unpaired t-test between two groups, and one-way analysis of variance (ANOVA) was used to perform comparison among more than two groups. Variables were analyzed at different time points using Bonferroni-corrected repeated measures ANOVA. All statistical analysis was completed with SPSS 21.0 software (IBM, Armonk, NY, USA), with two-tailed p < 0.05 as a level of statistical significance.

## Results

### Exosomes isolation from BMSCs

We aimed to clarify the function and mechanism of exosomes containing PLA, polylactic acid copolymer and BMP-2 in tendon bone healing of rotator cuff tear. Therefore, exosomes of PASP-PLGA microcapsules for sustained release of BMP-2 were selected for this study. First, BMSCs were isolated and purified to obtain exosomes. As shown in Figure 1a, all the rabbit BMSCs adhered to the wall and showed uniform spindle cell-like growth after subculture for 24 h. Flow cytometry showed that the rates of CD44 and CD90 positive cells were 93.4% and 90.4%, while rates of CD34 and CD45 negative cells were 5.58% and 9.21%, respectively (Figure 1b). These results demonstrated that BMSCs were successfully isolated and purified. TEM analysis showed that the isolated exosomes presented a typical exosomal double-layer capsule ultrastructure with saucer-shaped or hemispherical concave on one side (Figure 1c). NTA analysis showed that the peak particle diameter ranged from 100 to 200 nm with a mean ± SD of 112 ± 18 nm (Figure 1d). Flow cytometry analysis to CD9 and CD63 showed that CD9 and CD63 were highly expressed in the isolated exosomes (Figure 1e). We performed Western blots using targeting exosome markers, Alix, Annexin V, and TSG101, as well as a marker for contamination with cellular components, Calnexin. The results showed that Alix, Annexin V, TSG101 and Calnexin in the control group showed similar expression in the media group (figure 1f), which suggested the exosomes were successfully purified.

**Figure 1.** **Exosomes isolation from BMSCs**. (a) The morphology of BMSCs after subculture. Bar = 200 μm. (b) CD44, CD90 positive cells and CD34 and CD45 negative cells detected by flow cytometry. (c) Exosomes isolated from BMSCs detected by TEM. Bar = 1.0 μm. (d) Particle diameter of exosomes isolated from BMSCs detected by NTA analysis. (e) Flow cytometry analysis to CD9 and CD63 in the isolated exosomes of BMSCs. (f) Expression of exosome markers Alix, Annexin V, TSG101 and Calnexin detected by Western blot. GAPDH acted as control.

### Preparation of PASP-PLGA microcapsules for sustained release of BMP-2

We successfully established the PASP-PLGA microcapsules according to the technical route. By manipulating the process parameters, PASP-PLGA microcapsules with narrow size distributions (coefficient of variation was less than 15%), smooth morphology and various sizes, were obtained (Figure 2a). Encapsulation efficiency analysis showed that the encapsulation efficiency reached to >97% when we invested in PASP-PLGA microcapsules for 5, 10 and 20 mg BMP-2 (Figure 2b). Sustained release of BMP-2 tests in vitro showed that the microcapsules continuously released BMP-2, which could at least reach to 60 days (Figure 2c). The concentration of BMP-2 was also detected in the rabbit models of tendon-bone repair after an acute rotator cuff rupture at 4 weeks after treatment. The results showed that the concentration of BMP-2 was significantly elevated both in the serum and damaged tissue of rabbits (Figure 2d). These results demonstrated that the PASP-PLGA microcapsules sustainably released BMP-2.

**Figure 2.** **Preparation of PASP-PLGA microcapsules for sustained release of BMP-2**. (a) Technical route to establish the PASP-PLGA microcapsules. (b) Encapsulation efficiency analysis invest with in 5, 10 and 20 mg BMP-2 for PASP-PLGA microcapsules. All tests were repeated three times in triplicate. (c) Sustained release of BMP-2 tests in vitro. All tests were repeated three times in triplicate. (d) The concentration of BMP-2 was detected in the rabbit models of tendon-bone repair after acute rotator cuff rupture at 4 weeks after treatment. *p < 0.05 vs. control group. The data were expressed as mean ± standard deviation.

### Exosomes of PASP-PLGA microcapsules shows good stability and targeting

Exosomes of PASP-PLGA microcapsules were prepared by co-incubation of exosomes and PASP-PLGA microcapsules. TEM analysis showed that no significant changes in morphology of exosomes were observed after wrapping with PASP-PLGA microcapsules (Figure 3a). Meanwhile, the expression of exosome markers, Alix, Annexin V and Calnexin, did not present significant changes compared with the original exosomes as well (Figure 3b). In order to know the targeting characteristics of exosomes from PASP-PLGA microcapsules to BMSCs. The DiI-labeled exosomes of PASP-PLGA microcapsules were co-incubated with DiO labeled BMSCs. The results showed that the fluorescent signal was dramatically increased in the BMP-2-Exo groups compared with that in the Blank-Exo group and control-Exo groups (Figure 3c), suggesting that it was more conducive to ingest for BMSCs than exosomes in PASP-PLGA microcapsules. These results demonstrated that exosomes of PASP-PLGA microcapsules showed good stability and targeting of BMSCs.

**Figure 3.** **Exosomes of PASP-PLGA microcapsules showed good stability and targeting**. (a) TEM analysis to the changes of exosomes morphology after wrapping with PASP-PLGA microcapsules, Bar = 1.0 μm. (b) Expression of exosome markers Alix, Annexin V and Calnexin detected by Western blot. GAPDH acted as control. (c) The targeting characteristics of exosomes of PASP-PLGA microcapsules detected by DiI and Dio labeling. *p < 0.05 vs. control-Exo group. The data were expressed as mean ± standard deviation.

### Exosomes of PASP-PLGA microcapsules promotes tendon and bone interface healing after rotator cuff injury

To understand the function of exosomes of PASP-PLGA microcapsules in tendon and bone interface healing after rotator cuff injury, exosomes of PASP-PLGA microcapsules were used to treat tendon and bone interface after rotator cuff injury. Micro-CT was used to evaluate the effect of exosomes of PASP-PLGA microcapsules on microstructural properties of femurs. The results showed that exosomes of PASP-PLGA microcapsules promoted the tendon and bone interface healing after rotator cuff injury (Figure 4a). Further analysis showed that the BMD, TMD and BV/TV in the BMP-2 Exo group were significantly higher than those in the Control-Exo and Blank-Exo groups at 6, 12, and 18 weeks after surgery. And there were no significant differences in BMD, TMD and BV/TV between the Control-Exo and Blank-Exo group (Figure 4b–d). Furthermore, bone strength was determined by biomechanical tests. As shown in Figure 5, although the stiffness and the ultimate load strength of the tendon interface were impaired in the experimental group than that in the Sham group. However, the stiffness and the ultimate load strength of the tendon interface was significantly higher in BMP-2 Exo group than that in the Blank and Control-Exo groups at 6, 12, and 18 weeks after surgery.

**Figure 4.** **Micro-CT analysis to tendon and bone interface healing after treating with exosomes of PASP-PLGA microcapsules**. (a) Micro-CT was used to evaluate effects of exosomes of PASP-PLGA microcapsules on microstructural properties of femurs. n = 9. (b-d) The BMD, TMD and BV/TV of the BMP-2, Control-Exo and Blank-Exo groups at 6, 12, and 18 weeks after surgery, respectively. n = 9. **p < 0.01 vs. control-Exo group. The data were expressed as mean ± standard deviation.

**Figure 5.** **Stiffness and the ultimate load strength of the tendon bone interface was determined by biomechanical tests**. (a-b) Stiffness and the ultimate load strength of the tendon interface after treating with exosomes of PASP-PLGA microcapsules at 6, 12, and 18 weeks, respectively. **p < 0.01 vs. control-Exo group. The data were expressed as mean ± standard deviation.

In addition, we also performed histopathology analysis to evaluate the effect of exosomes of PASP-PLGA microcapsules on tendon and bone interface healing after rotator cuff injury. H&E analysis showed that inflammatory cells and visible capillary hyperplasia were observed in the Control-Exo and Blank-Exo groups. Fibrovascular granulation tissue filled the space between tendons and bones in the control group. Obvious bone ingrowth and chondrocytes were observed at the tendon–bone interface, and new fibrocartilage tissue began to appear in the BMP-2 group at 6 weeks after surgery. Inflammatory cells were reduced, and collagen fibers were increased at 12 weeks after surgery. The fibrocartilage tissue has not yet formed in the Blank-Exo and Control-Exo groups, while a larger area of bone tissue and fibrocartilage tissue formed in the BMP-2-Exo group. The inflammatory cells basically disappeared, and the collagen fibers at the tendon–bone interface were arranged neatly, all facing the direction of the tendon’s traction in the BMP-2-Exo group. The fibrocartilage tissue at the tendon–bone interface was remodeled to form a fibrocartilage layer, which was closer to the natural tendon-bone stop in BMP-2-Exo group (Figure 6a). Masson analysis showed that the collagen fibers were neatly arranged and distributed around the cartilage lacuna and the calcified cartilage and fibrocartilage combined tightly in the BMP-2-Exo group. However, collagen fibers were arranged in disorder, and the boundary between calcified cartilage and fibrocartilage fibers was unclear in the Control, Blank-Exo and Control-Exo groups at 18 weeks after treatment (Figure 6b). Alcian blue staining showed that chondrocytes were arranged in clusters at the bone healing boundary with darker staining in BMP-2-Exo group, while chondrocytes were sparse and inactive in the Control, Blank-Exo and Control-Exo groups at 18 weeks after treatment (Figure 6c). Taken together, these results indicated that exosomes of PASP-PLGA microcapsules promoted tendon and bone interface healing after rotator cuff injury.

**Figure 6.** **Histopathological changes of the tendon bone healing after treating with exosomes of PASP-PLGA microcapsules**. (a-c) HE, Masson and Alcian Blue staining to the tendon bone healing after treating with exosomes of PASP-PLGA microcapsules, respectively.

### Exosomes of PASP-PLGA microcapsules affects Smad/RUNX2 signaling pathway

In order to clarify which mechanism of exosomes of PASP-PLGA microcapsules participated in, BMSCs were treated with exosomes of PASP-PLGA microcapsules and the expression of several key proteins related to tendon regeneration was measured by immunofluorescence and Western blot, including CBFβ, TGFβ, Smad3, Smad4, Smad5, RUNX1, RUNX2 and Notch3. As shown in Figure 7a, the expressions of Smad4, Smad5 and RUNX2 were significantly increased when treated with exosomes of PASP-PLGA microcapsules, while no obvious changes were observed for the other genes. These results were also confirmed by Western blot (Figure 7b). In order to know the expression changes of Smad4, Smad5 and RUNX2 caused by BMP-2, the expression of BMP-2 was silenced by BMP-2 siRNA. The Western blot and immunofluorescence analysis showed that the expression of Smad4, Smad5 and RUNX2 was significantly decreased when silencing BMP-2 (Figure 7c,d). In addition, the expression and distribution of BMP-2, Smad4, Smad5 and RUNX2 were detected by immunohistochemistry and Western blot in rabbit models of tendon-bone repair after acute rotator cuff rupture. The immunohistochemistry analysis showed that BMP-2, Smad4, Smad5 and RUNX2 distributed throughout the bone tissue and the signaling of BMP-2, Smad4, Smad5 and RUNX2 were dramatically enhanced after treatment with exosomes of PASP-PLGA microcapsules (Figure 7e). Consistent with these results, Western blot analysis also indicated that the protein abundance of BMP-2, Smad4, Smad5 and RUNX2 was significantly increased after treatment with exosomes of PASP-PLGA microcapsules (Figure 7f). These results suggested that exosomes of PASP-PLGA microcapsules promoted tendon and bone interface healing after rotator cuff injury by regulating Smad/RUNX2 signaling pathway.

**Figure 7.** **Exosomes of PASP-PLGA microcapsules affected cartilage differentiation Smad/RUNX2 signaling pathway**. (a) The expression of CBFβ, TGFβ, Smad3, Smad4, Smad5, RUNX1, RUNX2 and Notch3 detected by immunofluorescence after treatment with exosomes of PASP-PLGA microcapsules. (b) The expression of CBFβ, TGFβ, Smad3, Smad4, Smad5, RUNX1, RUNX2 and Notch3 detected by Western blot after treatment with exosomes of PASP-PLGA microcapsules. (c) The expression of Smad4, Smad5 and RUNX2 was detected by immunofluorescence in BMP-2 silencing cells. (d) The expression of Smad4, Smad5 and RUNX2 was detected by Western blot in BMP-2 silencing cells. (e) The expression and distribution of BMP-2, Smad4, Smad5 and RUNX2 detected by immunohistochemistry after treatment with exosomes of PASP-PLGA microcapsules. (f) The expression of BMP-2, Smad4, Smad5 and RUNX2 detected by Western blot. GAPDH acted as control and the gray density calculated by ImageJ. **p < 0.01 vs. si-BMP2 group or control-Exo group. The data were expressed as mean ± standard deviation.

### Exosomes of PASP-PLGA microcapsules promotes cartilage differentiation via Smad/RUNX2 signaling pathway

Cartilage differentiation plays crucial roles in tendon and bone interface healing. Therefore, the expression of cartilage differentiation-related proteins was detected by Western blot and immunofluorescence in vitro, and Western blot and immunohistochemistry in vivo under treatment with exosomes of PASP-PLGA microcapsules, including Aggrecan, Collagen II, SOX-9 and TIMP-1. The expression of Aggrecan, Collagen II, SOX-9 and TIMP-1 was significantly elevated in both in vitro (Figure 8a,b) and vivo (Figure 8c,d) after treatment with exosomes of PASP-PLGA microcapsules. In order to understand the expression changes of these proteins affected by BMP-2, the expression of these proteins was detected by Western and immunofluorescence with BMP-2 knockdown in vitro. The results showed that the expression of Aggrecan, Collagen II, SOX-9 and TIMP-1 was significantly decreased when silencing BMP-2 (Figure 8e,f). These results indicated that exosomes of PASP-PLGA microcapsules might promote cartilage differentiation via Smad/RUNX2 signaling pathway.

**Figure 8.** **Exosomes of PASP-PLGA microcapsules affected cartilage differentiation via Smad/RUNX2 signaling pathway**. (a-b) The expression of Aggrecan, Collagen II, SOX-9 and TIMP-1 was detected by immunofluorescence and Western blot in vitro, respectively. (c-d) The expression of Aggrecan, Collagen II, SOX-9 and TIMP-1 was detected by immunohistochemistry and Western blot after treatment with exosomes of PASP-PLGA microcapsules in vivo, respectively. (e) The expression of Aggrecan, Collagen II, SOX-9 and TIMP-1 detected by immunofluorescence with BMP-2 knockdown in vitro. (f) The expression of Aggrecan, Collagen II, SOX-9 and TIMP-1 detected by Western blot with BMP-2 knockdown in vitro. **p < 0.01 vs. control-Exo group. The data were expressed as mean ± standard deviation.

## Discussion

In the present study, we successfully established the exosomes of PASP-PLGA microcapsules, which showed good stability and targeting. And we further demonstrated that exosome-delivered BMP-2 and PLA promoted tendon bone healing in rotator cuff tear via Smad/RUNX2 signaling pathway.

The histopathological manifestations of rotator cuff injury include cell structure destruction, tendon fiber thinning and structure disorders, granulation tissue hyperplasia and fibrocartilage degeneration [20,21]. Among them, the main problem is that the cartilage layer of the tendon–bone interface tissue cannot be regenerated, and it is only replaced by scar tissue, resulting in poor tendon bone healing. In recent years, various biological techniques have been used to promote the regeneration of cartilage at the tendon–bone interface after rotator cuff repair to restore the normal tissue morphology of the tendon-bone junction, improving mechanical performance and reducing post-operative tearing. Biological augmentation of rotator cuff repair provides new strategies to reinstate normal tendon bone structure, including cell growth factors, mesenchymal stem cells and biological enzymes. BMP-2, belonging to TGF family, has been indicated to play crucial roles in cartilage repair, extracellular matrix synthesis and chondrocyte differentiation [22–24], suggesting that BMP-2 might be used to heal tendon–bone in rotator cuff injury. However, it greatly restricts the application of BMP-2 in the treatment of rotator cuff injury due to the limited content of natural BMP-2, sustained release and unsustainable. So far, several studies have revealed that it promotes rotator cuff tendon-bone healing with injectable BMP-2 via different carriers, such as hyaluronic acid-coated gold nanorods, 10% poly(ethylene glycol) diacrylate (PEGDA) containing 0.05% of the photoinitiator and β-tricalcium phosphate [25–27]. Exosomes have become an efficient endogenous drug carrier for disease treatment, and it has also showed therapeutic potential of exosomes in rotator cuff tendon healing [28]. For example, macrophage-derived miRNA-containing exosomes induced peritendinous fibrosis after tendon injury through the miR-21-5p/smad7 pathway [15]. Exosomes isolated from adipose-derived stem cells can effectively decrease atrophy and degeneration and improve muscle regeneration and biomechanical properties in torn rotator cuff muscles [16,29]. Recently, a three-dimensional hydrogel comprised of BMP-2 core sequence oligopeptide, phosphoserine, a synthetic cell adhesion peptide (RGDS), and polyaspartic acid was found to synergistically promote osteogenesis performed, and in vitro experiments revealed that the peptide gel was conducive to adhesion and proliferation of rat marrow mesenchymal stem cells [18]. These results have provided the foundation to treat rotator cuff injury by combining the bone targeting properties of polyaspartic acid with the carrier function of exosomes, which can sustain release of BMP-2. In the present study, we successfully established exosomes of PASP-PLGA microcapsules and it sustained release BMP-2, which showed good stability and targeting to BMSCs. Further analysis showed that exosomes of PASP-PLGA microcapsules promoted tendon bone healing after rotator cuff injury. These results indicated that the new type of exosomes in PASP-PLGA microcapsules showed huge potential for the therapy of rotator cuff injury.

Several signaling pathways have been proved to involve in tendon bone healing, including Wnt/beta-Catenin, mTOR and Smad-RUNX2 pathways [30,31]. A number of biological processes can be regulated by Smad-RUNX2 signaling pathway, as well as osteoblastic differentiation. For example, vaspin antagonized high fat-induced bone loss in rats and promoted osteoblastic differentiation in primary rat osteoblasts through Smad-RUNX2 signaling pathway. Meanwhile, an increasing number of studies have demonstrated that the Smad/RUNX2 signaling pathway plays an important role in tendon bone healing in rotator cuff tear [19,32,33]. In addition, it has been demonstrated that BMP-2 can regulate osteogenic differentiation by affecting the expression of Smad and RUNX2. For example, BMP-2 enhanced osteogenic differentiation of stem cell spheres by regulation of RUNX2 expression. Melatonin rescued glucocorticoid-induced inhibition of osteoblast differentiation in MC3T3-E1 cells via the PI3K/AKT and BMP/Smad signaling pathways [34]. And it also has been showed that activation of the BMP-2-smad1/5/8 pathway enhances osteogenic differentiation of human bone marrow mesenchymal stem cells in ossification of the posterior longitudinal ligament [35]. However, few reports focus on whether Smad/RUNX2 signaling pathway participates in tendon bone healing regulated by BMP-2. In the present study, the expression of Smad4, Smad5 and RUNX2 was significantly increased when treated with exosomes of PASP-PLGA microcapsules, while the expression of Smad4, Smad5 and RUNX2 was significantly decreased when silencing BMP-2 both in vitro and in vivo. These results suggested that exosomes of PASP-PLGA microcapsules promoted tendon bone healing after rotator cuff injury by regulating the Smad/RUNX2 signaling pathway.

Several studies have showed that BMP-2 can participate in chondrogenic differentiation. For instance, Zhou et al. have demonstrated that BMP-2 induces chondrogenic differentiation, osteogenic differentiation and endochondral ossification in stem cells [36]. Mara et al. also have showed that rhBMP-2 increases chondrocyte proliferation, mineralization, and differentiation, suggesting that BMP-2 was required for postnatal maintenance of osteochondral tissues of the temporomandibular joint [37]. SIRT1 promoted BMP-2-induced chondrogenic differentiation of MSCs and reduced the apoptosis and decomposition of the extracellular matrix under oxidative stress [38]. It has also been demonstrated that BMP-2 delivery by coacervate and gene therapy can promote human muscle-derived stem cell-mediated articular cartilage repair [23]. In fact, studies have showed that cartilage differentiation plays crucial roles in tendon and bone interface healing [39]. These results suggest that BMP-2 regulates cartilage differentiation, which contributes to tendon bone interface healing. Aggrecan, Collagen II, SOX-9 and TIMP-1 have been proved as key factors contributing to cartilage differentiation. And these proteins also potentiate BMP-2-induced chondrogenic differentiation [40]. Consistent with these reports, the expression of cartilage differentiation-related proteins, Aggrecan, Collagen II, SOX-9 and TIMP-1, was significantly elevated both in vitro and in vivo after treatment with exosomes of PASP-PLGA microcapsules, while significantly decreased when silencing BMP-2. These results indicated that exosomes of PASP-PLGA microcapsules might affect cartilage differentiation via Smad/RUNX2 signaling pathway.

However, there were still some aspects that needed to be improved in our experimental design of animal models. In this study, only 2–3 samples per time point were evaluated for biomechanical evaluation, which was extremely low for biomechanical evaluation. In future study, biomechanical evaluation will be performed using more rabbit samples. Moreover, the signaling mechanism will be further explored by adding a group treated only with encapsulated BMP-2 on the basis of original grouping.

## Conclusion

In conclusion, we successfully established the exosomes of PASP-PLGA microcapsules, which showed good stability and targeting. Function and mechanism analysis of the exosomes of PASP-PLGA microcapsules demonstrated that exosome-delivered BMP-2 and PLA promote tendon bone healing in rotator cuff tear via Smad/RUNX2 signaling pathway. These findings may provide a new idea for promoting tendon healing and provide a basis to explore the further application potential of this bioactive scaffold.

## Data Availability

The datasets during and/or analyzed during the current study are available from the corresponding authors on reasonable requests.

## Article highlights

- Exosomes of PASP-PLGA microcapsules showed good stability and targeting.
- Exosomes of PASP-PLGA microcapsules promoted tendon and bone interface healing after rotator cuff injury.
- Exosomes of PASP-PLGA microcapsules affected Smad/RUNX2 signaling pathway.
- Exosomes of PASP-PLGA microcapsules promoted cartilage differentiation via Smad/RUNX2 signaling pathway.
